This article has been retracted.

# Causal relationship between dyslipidemia and risk of facial aging: Insights from Mendelian randomization in East Asian populations

**DOI:** 10.1111/srt.13717

**Published:** 2024-05-08

**Authors:** Yu Deng, Chuan Li, Ailin Luo, Yang Qiu, Mei Yang

**Affiliations:** ^1^ Department of Thoracic Surgery West China Hospital, Sichuan University Chengdu Sichuan China

**Keywords:** dyslipidemia, East Asian, facial aging, high‐density‐lipoprotein cholesterol, Mendelian randomization

## Abstract

**Background:**

Emerging observational studies showed an association between dyslipidemia and aging. However, it remains unclear whether this association is causal, particularly in the case of Asians, which are aging more rapidly than other continents. Given the visible manifestations of aging often include changes in facial appearance, the objective of this study is to assess the causal relationship between dyslipidemia and facial aging in East Asian populations.

**Methods:**

SNPs related to dyslipidemia in East Asian people such as Total cholesterol (TC), High‐density‐lipoprotein cholesterol (HDL), Low‐density‐lipoprotein cholesterol (LDL), and Triglyceride (TG) along with outcomes data on facial aging, were extracted from public genome‐wide association studies (GWAS). A two‐sample Mendelian randomization (MR) analysis was then performed using publicly available GWAS data to investigate the potential causal relationship. The effect estimates were primarily calculated using the fixed‐effects inverse variance weighted (IVW) method.

**Results:**

Totally, 88 SNPs related to HDL among 70657 East Asian participants in GWAS. Based on the primary causal effects model using MR analyses with the IVW method, high HDL level was demonstrated as significantly related to the risk of facial aging (OR, 1.060; 95% CI, 1.005–1.119, *p* = 0.034), while high TC level (OR, 0.995; 95% CI, 0.920–1.076, *p* = 0.903), high LDL level (OR, 0.980, 95% CI, 0.924–1.041, *p* = 0.515), as well as high TG level (OR, 0.999, 95% CI, 0.932–1.071, *p* = 0.974), showed no significant correlation with facial aging.

**Conclusions:**

The two‐sample MR analysis conducted in this study revealed a positive causal relationship between high HDL levels and facial aging. In contrast, facial aging demonstrated no significant correlation with high levels of TC, LDL, or TG. Further large‐sample prospective studies are needed to validate these findings and to provide appropriate recommendations regarding nutrition management to delay the aging process among old patients in East Asia.

## 1 INTRODUCTION

Dyslipidemia, characterized by abnormal lipid levels in the bloodstream, is commonly associated with various cardiovascular risks.^1^ However, its relationship with facial aging, a complex process influenced by both genetic and environmental factors, is not as straightforward. Facial aging involves changes in skin elasticity, wrinkle formation, and collagen degradation.^2^ Studies have suggested that dyslipidemia may exacerbate these aging processes due to the impact of lipids on skin integrity and inflammation.^3^ Conversely, other research points to a lack of direct correlation between dyslipidemia and accelerated facial aging, indicating that factors such as UV exposure and lifestyle choices play a more significant role.^4^, ^5^ Thus, the current understanding of the link between dyslipidemia and facial aging is inconclusive and marked by contradictions. Further investigation is needed to clarify this relationship, considering the potential influence of other variables such as dietary habits and genetic predisposition, to develop a more comprehensive understanding of how dyslipidemia might affect facial aging.

Mendelian randomization (MR) has emerged as a prominent method for examining the potential causative links between various exposures and health outcomes.^6^ Differing from traditional observational research, MR analysis uniquely counters reverse causation bias, given that the random allocation of alleles happens prior to the development of diseases. This methodology leverages the random distribution and independent assortment of genetic variations at the time of conception. By employing genetic markers as instrumental variables (IVs), MR effectively reduces the impact of confounders.^7^, ^8^ The widespread availability of comprehensive genome‐wide association studies (GWASs) enhances the capacity for causal investigations. Utilizing MR analysis, this study seeks to unravel a critical inquiry: What is the nature of the relationship between Dyslipidemia and Facial aging‐is it negative, neutral, or positive?

## 2 MATERIALS AND METHODS

### 2.1 Study design

Figure 1 depicts the research methodology, highlighting MR's three core hypotheses: (A) Significant correlation between single nucleotide polymorphisms (SNPs) and lipid profiles, including Total cholesterol (TC), High‐density‐lipoprotein cholesterol (HDL), Low‐density‐lipoprotein cholesterol (LDL), and Triglycerides (TCG); (B) SNPs' autonomy from established confounding variables; and (C) The exclusive influence of SNPs on Facial aging is channeled through lipid levels such as TC, HDL, LDL, and TCG.^9^

**FIGURE 1:** The fundamental assumptions of the Mendelian randomization study: (A) Single‐nucleotide polymorphisms (SNPs) have a strong association with TC, HDL, LDL, and TG; (B) SNPs are not influenced by confounding factors; (C) SNPs impact facial aging exclusively through TC, HDL, LDL, and TG. TC, Total cholesterol; HDL, high density lipoprotein; LDL, low density lipoprotein; TG, Triglyceride.

### 2.2 Data sources

The study conducted a comprehensive analysis using open‐access, summary‐level data from GWASs, which predominantly targeted traits in East Asian populations, including both genders. The research specifically extracted GWAS summary data for Total cholesterol (128305 participants), HDL (70657 participants), LDL (72866 participants), and Triglycerides (105597 participants) from findings by Ishigaki K, examining the link between dyslipidemia and single nucleotide polymorphisms (SNPs). Additionally, data on Facial aging (GWAS ID: ukb‐e‐1757_EAS, involving 2530 individuals) was sourced from the Pan‐UKB team's investigation, which identified 8255761 SNPs related to the study (Table 1). Given that all GWAS datasets used in this analysis are readily accessible and have received prior approval from respective ethical review boards, obtaining fresh ethics approval for this study was deemed unnecessary.

**TABLE 1:** The characteristics of GWAS data.

Trait	Sample size	GWAS ID	Year	author	Population	n SNP
Total cholesterol	128305	bbj‐a‐54	2019	Ishigaki K	East Asian	6108953
HDL	70657	bbj‐a‐24	2019	Ishigaki K	East Asian	6108953
LDL	72866	bbj‐a‐31	2019	Ishigaki K	East Asian	6108953
Triglyceride	105597	bbj‐a‐55	2019	Ishigaki K	East Asian	6108953
Facial aging	2530	ukb‐e‐1757_EAS	2020	Pan‐UKB team	East Asian	8255761

Abbreviations: GWAS, genome‐wide association studies; HDL, high density lipoprotein; LDL, low density lipoprotein; SNP, single‐nucleotide polymorphism.

### 2.3 Selection and validation of SNPs

To select suitable SNPs, three distinct criteria were applied. First, SNPs linked to TC, HDL, LDL, and TCG were pinpointed, meeting the genome‐wide significance threshold (*p* < 1 × 10^–5^). Next, the independence of these SNPs was ascertained by analyzing pairwise‐linkage disequilibrium.^10^ Any SNP with an r2 greater than 0.001, within a 10000 kb clumping window, was excluded if it demonstrated high correlation with multiple SNPs or possessed a larger *p*‐value. The third step involved calculating the F‐statistic to determine the individual strength of each SNP. Those with an F‐statistic exceeding ten were deemed strong enough to minimize potential bias.^11^ Prior to initiating the MR analysis, we conducted data‐harmonization procedures to ensure that the effects attributed to an SNP on both the exposure and the outcome were aligned with the same allele.

### 2.4 MR analysis

The main analysis incorporated an inverse‐variance weighted (IVW) meta‐analysis utilizing a fixed‐effects approach. To examine pleiotropy, the MR‐PRESSO method was employed, aiding in the assessment of horizontal pleiotropy in the chosen IVs.^12^ Cochrane's Q‐value served as the metric for gauging heterogeneity among these IVs. Additionally, a leave‐one‐out sensitivity analysis was executed to determine the influence of individual SNPs on the aggregate results. All statistical evaluations were carried out using the “TwoSampleMR” package within R version 4.0.3, as provided by the R Foundation for Statistical Computing in Vienna, Austria.

## 3 RESULTS

### 3.1 SNP selection and validation

To summarize, the research incorporated in our analysis was conducted between 2019 and 2020, with a primary emphasis on the East Asian demographic (referenced in Table 1). Each of the chosen IVs achieved genome‐wide significance, and all exhibited F‐statistics exceeding ten (as detailed in Table 2).

**TABLE 2:** Single nucleotide polymorphisms used as instrumental variables in the Mendelian randomization analyses of HDL.

SNP	Chr	EA	NEA	Beta	SE	F
rs10066035	5	T	C	−0.02672	0.005517	23.45670142
rs1011223	16	A	G	0.05068	0.00908	31.15311766
rs1026422	7	A	G	0.03266	0.005247	38.74451532
rs10774684	12	T	C	−0.02711	0.005421	25.00922424
rs10793129	11	A	G	−0.03438	0.00614	31.35270401
rs10820720	9	C	A	−0.02531	0.005231	23.41072429
rs11057855	12	G	A	0.04848	0.009421	26.48080692
rs11079285	17	T	C	−0.02887	0.006324	20.84058211
rs11082764	18	G	A	0.07838	0.005219	225.546413
rs11102000	1	C	G	0.02632	0.005822	20.43748107
rs11177683	12	A	G	−0.02419	0.005463	19.60691814
rs11657865	17	C	A	0.02724	0.005303	26.38584168
rs117350179	3	G	C	−0.0343	0.006187	30.73463133
rs1204834	6	A	T	−0.02582	0.005466	22.31378382
rs12293222	11	A	G	−0.06562	0.005454	144.7578702
rs1243668	14	T	C	0.02954	0.006646	19.75605871
rs12516382	5	A	G	−0.02878	0.005318	29.28767612
rs12547186	8	A	G	−0.0261	0.005711	20.88606832
rs1358980	6	T	C	−0.0313	0.005261	35.39582763
rs17369578	16	A	G	0.06359	0.00885	51.62869035
rs1883025	9	T	C	−0.1081	0.00585	341.4598583
rs2043082	15	A	G	0.1146	0.005277	471.6230764
rs2070895	15	A	G	0.1322	0.005235	637.719267
rs2144300	1	T	C	0.03663	0.006685	30.02417026
rs2257129	10	C	T	−0.0365	0.005727	40.61919972
rs2278986	12	G	A	−0.03622	0.006997	26.7961959
rs2297409	9	A	G	−0.04587	0.005382	72.63903958
rs235314	21	T	C	−0.03324	0.00529	39.4830493
rs2487032	9	A	G	0.02368	0.005243	20.39875588
rs2642438	1	G	A	0.03094	0.007004	19.51409181
rs2655167	8	T	C	−0.03377	0.007379	20.94436031
rs2714876	7	A	C	−0.02606	0.005586	21.76441308
rs28366301	6	A	G	0.03687	0.005664	42.37403157
rs2925979	16	C	T	0.03966	0.00553	51.43457518
rs2954038	8	A	C	0.03129	0.005822	28.88462437
rs325	8	C	T	0.1483	0.007858	356.1707519
rs333968	1	T	C	−0.03282	0.006183	28.175956
rs34287007	13	C	G	0.1148	0.02506	20.98561218
rs34398286	4	T	C	0.02965	0.00628	22.29102854
rs3753312	1	A	C	−0.03001	0.006678	20.19478163
rs3768320	1	C	T	0.03637	0.00718	25.65888106
rs3808447	8	A	G	0.04848	0.006163	61.87865808
rs3858704	12	G	A	0.08707	0.005555	245.6795242
rs4140856	8	G	A	−0.03343	0.007344	20.72084284
rs41437847	12	G	A	−0.03742	0.006588	32.2626759
rs4149310	9	T	A	0.06261	0.00567	121.9330086
rs429358	19	C	T	−0.08948	0.00879	103.6273043
rs4752898	11	C	T	−0.1028	0.02243	21.00524165
rs4765153	12	T	C	0.05077	0.008979	31.97115925
rs4805010	19	A	C	0.02453	0.005525	19.71199279
rs4917630	10	A	G	−0.03894	0.005432	51.38926093
rs4938293	11	T	C	−0.03313	0.005666	34.1892624
rs55723461	15	G	T	0.05447	0.005381	102.4681196
rs56156922	16	C	T	0.2656	0.006444	1698.811053
rs56303487	16	T	C	0.06921	0.007719	80.39251524
rs57947200	2	A	T	−0.05389	0.01004	28.81037702
rs59156491	11	T	C	0.03113	0.005514	31.87313027
rs61863116	10	G	A	−0.0321	0.006067	27.99381414
rs61971506	14	A	G	0.03337	0.00684	23.80127432
rs662799	11	A	G	0.143	0.00541	698.6787663
rs6685271	1	A	C	−0.0387	0.006028	41.21691122
rs6687315	1	A	G	−0.02872	0.005931	23.44838969
rs67053123	12	A	T	0.07064	0.005942	141.3305621
rs6782707	3	A	T	−0.0298	0.006706	19.74719569
rs6991199	8	A	G	−0.02679	0.005331	25.25387707
rs72642493	18	C	A	0.0451	0.007163	39.64269594
rs72739195	15	C	T	0.06908	0.007897	76.52095505
rs72759626	1	C	T	−0.03093	0.006524	22.47666824
rs72773120	16	T	C	−0.1018	0.007825	169.2492931
rs7295954	12	T	C	−0.06478	0.01052	37.91843528
rs7307039	12	G	A	0.0411	0.005967	47.44293716
rs7310944	12	A	G	−0.04945	0.005465	81.8751784
rs74246262	16	T	G	0.1557	0.01238	158.1743053
rs7445	22	T	C	−0.04087	0.0053	59.46446778
rs76083992	20	T	C	−0.08508	0.01123	57.39782687
rs769446	19	C	T	0.08315	0.0134	38.50480341
rs7778167	7	A	G	0.05556	0.008285	44.97171488
rs7847628	9	G	A	−0.03203	0.005671	31.90028644
rs7895716	10	G	C	0.0353	0.005487	41.38848126
rs7938710	11	T	C	−0.0312	0.006744	21.40297109
rs79439130	20	A	G	0.04618	0.008731	27.97563034
rs79719909	12	G	A	0.0375	0.007874	22.68149698
rs80189144	7	C	T	0.04558	0.008903	26.21053556
rs8030365	15	A	G	−0.02656	0.005783	21.09355389
rs886479	12	C	A	0.05166	0.00538	92.20283025
rs889606	16	G	C	0.03218	0.00679	22.46117807
rs9304644	19	T	C	0.03438	0.005494	39.15925624
rs940541	7	G	A	−0.04066	0.00689	34.82541535

Abbreviations: Chr, chromosome; EA, effect allele; HDL, high density lipoprotein; NEA, non‐effect allele; SE, standard error; SNP, single nucleotide polymorphisms.

### 3.2 Total cholesterol and facial aging

The IVW approach indicated no significant association between TC levels and Facial aging (Odds Ratio [OR], 0.995; 95% Confidence Interval [CI], 0.920–1.076; *p* = 0.903). Consistent with IVW findings, both MR Egger and weighted median methods produced similar outcomes (OR, 0.927; 95% CI, 0.810–1.060; *p* = 0.269 and OR, 0.910; 95% CI, 0.807–1.026; *p* = 0.122, respectively) (Figure 2). These analyses showed no signs of heterogeneity (*p* = 0.690) or horizontal pleiotropy (*p* = 0.661), as detailed in Table 3. Additionally, the leave‐one‐out sensitivity analysis, illustrated in Figure S1, affirmed that the results were not disproportionately influenced by any single SNP.

**FIGURE 2:** The relationships between genetically predicted levels of total cholesterol, HDL, LDL, and Triglyceride, and their effects on facial aging. CI, confidence interval; HDL, high density lipoprotein; LDL, low density lipoprotein; OR, odds ratio.

**TABLE 3:** The result of heterogeneity and pleiotropy test.

Exposes	Heterogeneity		Pleiotropy	
	Q	*p*	RSSobs	*p*
Total cholesterol	70.346	0.690	74.171	0.661
HDL	71.755	0.880	73.572	0.877
LDL	38.338	0.947	43.769	0.911
Triglyceride	64.992	0.871	66.687	0.882

Abbreviations: HDL, high density lipoprotein; LDL, low density lipoprotein.

### 3.3 HDL and facial aging

In the primary analysis of causal effects using MR with the IVW method, a notable correlation was observed between elevated HDL levels and the risk of Facial aging (OR, 1.060; 95% CI, 1.005–1.119; *p* = 0.034, as seen in Figure 2). However, alternative methods like MR‐Egger (OR, 1.041; 95% CI, 0.949–1.141; *p* = 0.401) and weighted median (OR, 1.023; 95% CI, 0.937–1.118; *p* = 0.611) did not establish a statistically significant link between HDL levels and Facial aging, yet their effect direction was consistent with the IVW method. The absence of potential heterogeneity was confirmed through heterogeneity analysis (*p* = 0.880, Table 3), enhancing the credibility of the IVW findings. Additionally, the MR results showed no signs of horizontal pleiotropy (*p* = 0.877). Both the forest plot and scatter plot, depicted in Figure 3 and Figure 4 respectively, underscored the consistency of these results. The leave‐one‐out sensitivity analysis, illustrated in Figure S1, verified that no single SNP disproportionately impacted the overall estimates.

**FIGURE 3:** Forest plot of the association of HDL and Facial aging. HDL, high density lipoprotein.

**FIGURE 4:** Scatter plot of the association of HDL and Facial aging. HDL, high density lipoprotein.

### 3.4 LDL and facial aging

The application of the IVW method revealed no significant link between LDL levels and Facial aging (OR, 0.980; 95% CI, 0.924–1.041; *p* = 0.515). This finding was echoed in the MR Egger and weighted median analyses, which showed ORs of 0.924 (95% CI, 0.853–1.001; *p* = 0.060) and 0.927 (95% CI, 0.856–1.004; *p* = 0.064), respectively (Figure 2). Notably, heterogeneity tests indicated no substantial heterogeneity (*p* = 0.947), enhancing the trustworthiness of these outcomes. Moreover, the MR‐PRESSO intercept analysis found no evidence of directional pleiotropy (*p* = 0.911), as documented in Table 3. Sensitivity analyses, illustrated in Figures S1 and S2, further corroborated that the collective estimates were not significantly skewed by any individual SNP.

### 3.5 Triglyceride and facial aging

The MR analyses consistently demonstrated that TCG did not exhibit a significant genetic association with Facial aging, as evidenced by the following results: OR of 0.999 (95% CI, 0.932–1.071; *p* = 0.974) for IVW, OR of 1.043 (95% CI, 0.935–1.164; *p* = 0.453) for MR Egger, and OR of 0.982 (95% CI, 0.878–1.098; *p* = 0.748) for the weighted median approach (Figure 2). Furthermore, these analyses found no indications of heterogeneity (*p* = 0.871) or horizontal pleiotropy (*p* = 0.882), as detailed in Table 3. The leave‐one‐out sensitivity analysis, illustrated in Figure S1, confirmed that the aggregate results were not disproportionately affected by any single SNP.

## 4 DISCUSSION

In recent aging research, the influence of dyslipidemia, defined by irregular levels of lipids in the blood, on facial aging has become a topic of significant interest.^13^ While prior research has examined this link, findings have been mixed, with some studies not finding a definitive connection between dyslipidemia and the aging of facial features.^4^ In light of this, our study focuses on dyslipidemia as a key element, utilizing MR to delve into its association with facial aging. The MR approach allows for the assessment of a cause‐and‐effect relationship between dyslipidemia and facial aging, using genetic variations as IVs, which helps to reduce the bias usually seen in observational studies.^14^

This study represents the inaugural use of MR to investigate the causal impact of dyslipidemia on facial aging. Utilizing a two‐sample MR approach, we conducted an extensive analysis to understand the causal links between various lipid profiles—TC, HDL, LDL, and TCG—and the aging of facial features. Our findings indicate a casual correlation where elevated HDL levels could contribute to an increased risk of facial aging. This aligns with the observations made by Johanna et al. in 2019, who also noted a heightened risk of age‐related diseases in individuals with higher HDL levels.^15^ Notably, our MR methodology provides more robust conclusions than prior observational studies, given its resistance to confounding variables and avoidance of reverse causality.

There are several possible mechanisms that could explain the causal relationship between the elevated HDL levels and the development of facial aging: (1) Antioxidant Effects: HDL has antioxidant properties. While this is generally positive, a high level of antioxidants might interfere with certain cellular processes. In skin aging, the balance between oxidative stress and antioxidant defense is crucial. Overabundance of antioxidants could disrupt this balance, potentially affecting skin aging.^16^ (2) Influence on Skin Lipids: HDL plays a role in lipid metabolism. Changes in the lipid composition of the skin can influence skin barrier function and hydration, which are critical in maintaining youthful skin. Excessive or altered HDL levels might disrupt the normal lipid balance in the skin, leading to changes associated with aging.^17^ (3) Impact on Hormonal Balance: Lipoproteins can influence hormonal levels and metabolism. Hormones like estrogen have a known impact on skin health and aging. Elevated HDL might indirectly affect facial aging through hormonal pathways.^18^ (4) Modulation of Inflammation: Although HDL is typically anti‐inflammatory, the role of inflammation in aging (including skin aging) is complex. It's possible that changes in inflammatory responses due to altered HDL levels could accelerate aging processes in the skin.^19^

Our study confirmed a causal relationship between the elevated HDL levels and the acceleration of facial aging, which has important implications for clinical practice and prevention strategies. The following are possible clinical applications: (1) Preventive Healthcare: Patients with naturally high HDL levels or those taking medication to increase HDL might be monitored more closely for signs of accelerated facial aging. This could lead to early intervention strategies. (2) Aesthetic and Dermatological Treatments: This knowledge can guide dermatologists and cosmetic surgeons in advising patients who are concerned about facial aging. For those with elevated HDL levels, specific anti‐aging treatments could be recommended. (3) Nutritional Advice: Since HDL levels can be influenced by diet, nutritionists could use this information to give advice that balances cardiovascular benefits with potential impacts on facial aging.

This study presents various strengths and limitations. Its primary strength is the use of MR analysis, which minimizes biases related to residual confounding and reverse causation. This approach significantly bolsters the thorough investigation of the HDL‐facial aging relationship. However, several constraints need acknowledgment. Firstly, completely ruling out the impact of directional pleiotropy in MR studies is inherently difficult. Nonetheless, our MR‐PRESSO assessments found no pleiotropic effects, and our sensitivity analyses yielded consistent findings. Secondly, the GWASs we reviewed primarily involved East Asian individuals, which may limit the applicability of our results to other ethnic groups. Lastly, the lack of detailed data on the types of HDL restricted our ability to explore variations in the association with HDL levels based on these specific characteristics.

This two‐sample MR analysis found a causally positive association between HDL level and facial aging, suggesting that higher levels of HDL, commonly known as “good cholesterol,” might be linked to increased signs of aging in the face. The implications of this finding are multifaceted, as HDL is typically associated with various health benefits, particularly in terms of cardiovascular health. However, this research introduces a novel perspective by possibly linking it to an aging or dermatological outcome.

## CONFLICT OF INTEREST STATEMENT

No disclosures were reported.

## Supporting information

Supporting Information

Supporting Information

Supporting Information

## Data Availability

The datasets used in this study are available from the corresponding author upon reasonable request.
